# Analysis of Pathogen Characteristics and Nursing Factors of Tonsil Infection Based on Regression Equation

**DOI:** 10.1155/2022/3149619

**Published:** 2022-06-11

**Authors:** Longfang Zhang, Yuanyuan Yang

**Affiliations:** Department of Otorhinolaryngology and Stomatology, The First Affiliated Hospital of Soochow University, Suzhou, Jiangsu 215008, China

## Abstract

In order to meet the needs of the analysis and application of regression equation in clinical medicine of tonsil infection, this paper focuses on the semiparametric regression model method, cross-validation method, empirical method, and multiple regression equation analysis of atypical data using regression equation. The general method of analyzing this kind of data is given, and the parameter estimation and hypothesis testing of the model are systematically studied. The experimental results showed that among the 90 paraffin-embedded tissue specimens of chronic tonsillitis and adenoid hypertrophy in this study, 26 out of 49 male children were EBERs positive, accounting for 53.06% of male children (26/49 cases). 28 of the 41 female children were positive, accounting for 68.29 of the female children (28/41 cases). There were 14 cases in infant group, 20 cases in preschool age group, 25 cases in school-age group, and 31 cases in adolescence group; the EBERs-positive rate was 42.86% (6/14 cases) in early childhood and 55.00% in early school-age (11/20 cases), and the EBERs-positive rate was 60.00% in school-age group (15/20 cases) and 70.97% in adolescent group. The results showed that the latent infection rate of adenoid hypertrophy EBV in children with chronic tonsillitis showed no significant difference between genders. It is proved that the regression equation method can meet the needs of clinical analysis and application of tonsil infection.

## 1. Introduction

Tonsillitis is a very common disease that is rarely considered an important risk factor for oropharyngeal cancer, but the relationship between inflammation and carcinogenesis has been well documented. Foreign scholars have also confirmed that there is a correlation between the development of nasopharyngeal carcinoma and surrounding inflammation [1]. Although inflammatory processes are known to increase the risk of cancer, the relationship between chronic tonsillitis and cancer remains unknown. High-risk HPV and EBV infection play an important role in tumor transformation of human oral epithelial cells, and viral infection does play a role in inducing cancer mechanism, but the potential role of viral infection leading to virus-induced carcinogenesis has not been verified [2]. As a simple and effective method to find the regression equation, the least square method has been mastered and widely used. Recent studies on the robustness of mathematical statistics have found that when there are out varies, the robustness of the regression equation obtained by the least square method is often affected [3]. In this regard, some methods of robust regression are proposed to overcome this defect. For example, a more robust regression equation can be obtained by using the absolute sum of residuals as the objective function of minimization, that is, the least one method; see Figure 1 [4]. In this paper, by using the robustness of median over mean, and with the aid of residual analysis, a new robust regression equation is presented to analyze the characteristics of tonsillar infection pathogens and nursing factors that can resist the interference of abnormal data by several iterations of the initial regression equation.

## 2. Literature Review

Wang and Zhang believed that the parameter estimation of multiple regression models in previous studies usually adopts the least square parameter estimation method, but the least square regression model requires no collinearity between independent variables. When there is serious collinearity between independent variables, the parameter estimation will be seriously harmed, the model error will be increased, and the robustness of the model will be destroyed. In addition, multiple linear regression often requires the sample content to be 10~20 times of the number of variables. In practical problems, it is sometimes difficult to expand the sample content [5]. To solve this problem, Undiyaundeye proposed a new multivariate statistical analysis method partial least squares (PLS) regression in 1983 [6]. Grauso et al. has studied and pointed out that in the regression modeling of dependent variable to multiple independent variables, when there is a high degree of correlation within each variable set, the partial least squares regression modeling analysis is more effective than the general multiple regression, and its conclusion is more reliable [7]. By analyzing the function of partial least squares regression on the synthesis and screening of multivariate information, Attafuah et al. revealed the modeling mechanism of partial least squares regression under multiple correlation conditions and also demonstrated the extensive application scope of this new multivariate analysis method [8]. Yu et al. used specific examples to compare and analyze the least squares regression (MLR) principal component regression (PCR) and partial least squares regression (PLS), revealing that PLS can provide a more reasonable. In addition to the robust regression model, some research contents similar to principal component analysis and canonical correlation analysis can be completed at the same time to provide more rich and in-depth information [9]. Lu et al. believes that partial least squares regression analysis provides a many-to-many linear regression modeling method to establish linear or even nonlinear regression prediction equations of dependent variables with respect to independent variables. It is especially suitable for the case where two groups of variables have a large number of multiple correlations and the amount of observed data is small [10]. Bazan et al. believed that the least square regression analysis was initially applied in the field of metrology and achieved success. In recent years, it has been rapidly extended to other fields, such as bioinformatics and social sciences, and achieved good results. However, it is seldomly applied in the field of medicine and health, which explains the application analysis of partial least square regression of tonsil infection pathogen characteristics and nursing influencing factors [11]. Tarr et al. noted that with the deepening understanding of disease and its influencing factors and various indicators, multifactor analysis method has been widely used. Multivariate analysis, also known as multivariate statistical analysis, is a series of statistical methods to study the relationship between multiple factors (variables) and the relationship between samples (individuals) with these factors, such as discriminant analysis, cluster analysis, and principal component analysis [12]. In this series of methods, multivariate linear regression is the basis of multivariate statistical methods to study the linear relationship between multiple independent variables and one dependent variable.

On the basis of the current research, this paper focuses on the semiparametric regression model method, cross-validation method, empirical method, and multiple regression equation analysis of atypical data by using regression equation; gives the general method of analyzing this kind of data; and systematically studies the parameter estimation and hypothesis testing of the model, to prove the effect of regression equation method on clinical analysis and application of tonsil infection.

## 3. Research Method

### 3.1. Semiparametric Regression Model Method

In practical problems, people often encounter other situations where the assumptions of the classical statistical model cannot be fully satisfied. For example, the specific dependency relationship between response variables and explanatory variables is not clear or linear; that is, the model formal assumption does not meet the distribution of response variables, is not easy to judge, or does not meet the required distribution, that is, the data source assumption does not meet. At this point, the classical regression analysis method cannot guarantee good results, parameter estimates are unreliable, and it is even difficult to give a reasonable explanation for the selling problem. Therefore, classical statistical methods have their limitations; it is difficult to conduct regression analysis on atypical data, while nonparametric regression, one of the exploratory analysis methods, can effectively analyze atypical data.

At this point, the classical regression analysis method cannot guarantee good results. Parameter estimates are not reliable, and it is even difficult to give a reasonable explanation of the sellability problem. Therefore, classical statistical methods have their limitations. It is difficult to perform regression analysis on atypical data, but nonparametric regression, one of the exploratory analysis methods, can effectively analyze atypical data [13].

According to the different assumptions of regression function, regression models can be divided into two types: parametric regression model and nonparametric regression model. If the regression function belongs to a class of functions determined by a finite number of parameters, the function form is known, and the parameters are unknown, that is, the model form is known, and it is called parametric regression model. If the regression function is restricted to a certain class of smooth functions, such as continuously differentiable functions with square integrable second derivatives, that is, a set of functions belonging to an infinite dimension, it is called a nonparametric regression model. Like classical regression, nonparametric regression also has two main purposes: one is to explore and describe the relationship between variables, and the other is to predict and estimate, that is, regression is regarded as a model-based data induction method [14].

The model studies the dependence between the response variable and the single explanatory variable *t*, and it can solve many important problems. However, in practical work, many things or phenomena are affected by multiple variables, so it is necessary to study the relationship between multiple variables. Multiple regressions are often used in statistical analysis to study the dependence relationship affected by multiple explanatory variables, and the more general model of multiple regressions is the linear model: *y*_*i*_ = *x*_*i*_′*β* + *ε*_*i*_. *x*_*i*_ is the vector composed of the *i*th observed explanatory variable, which can be a continuous variable or a categorical variable. *β* is the unknown regression coefficient vector. In general, *x*_*i*_ contains a constant *L* corresponding to the intercept [15]. In order to relax the linearity assumption of one of the explanatory variables in the linear model, a semiparametric regression model can be considered.

#### 3.1.1. Model Description

Assume that for each observation *y*_*i*_, there is a *p* + 1 explanatory variable, in which the *p*-dimensional vector *x*_*i*_ and the quantitative variable *t*, and if the reaction variable *y* is linearly related to the explanatory variable *x*, there is the following model, as

(1) $$\begin{array}{c} y_{i}=x_{i}^{\text{'}}\beta +g\left(t_{i}\right)+\varepsilon_{i} \end{array}$$

is an unknown *p*-dimensional regression coefficient vector *β*, *g* (*t*) is an unknown smooth function, *x* is a linear variable, and *t* is a spline variable. *ε* is independent of delta (*x*, *y*). *E* (*ε*) = 0, and *V* (*ε*) = *σ*^2^ (unknown). Obviously, *x*_*i*_ does not contain constant *l*, and the constant term can be included in *g*(*t*), so the above model is called semiparametric regression model or partial spline.

The semiparametric regression model is more adaptable than the parametric linear model. In practical work, the semiparametric regression model is an extension of the linear model because some variable often has an influence on the performance of the unknown function. In the actual application of Model Formula (1), response variables are linearly correlated, and most explanatory variables should be based on professional theoretical knowledge or previous experience. The processing of spline *T* variable is different from other linear variables in that it is processed in a nonparametric form.

The semiparametric regression model is solved by the penalty least squares method, where the estimation of *β* and *g*(*t*) minimizes the following weighted sum of penalty squares.

(2) $$\begin{array}{c} S_{w}\left(\beta ,g\right)=\overset{n}{\underset{t=1}{\sum }}w_{i}{\left\{y_{i}-x_{i}^{\text{'}}\beta -g\left(t_{i}\right)\right\}}^{2}+\alpha \int g^{\prime \prime }{\left(t\right)}^{2}dt. \end{array}$$

Smooth parameter *α* > 0, *w*_*i*_ > 0, and *w*_*i*_ = 1 without weighting [16].

Set *Y* = (*y*_l_ ⋯ *y*_*n*_)′, *W* = diag(*w*_*i*_, ⋯, w_n_), *X* is *n*∗*p* n-matrixn, the *i*th is *x*_*i*_′; to consider the stalemate, suppose *t*_1_, t_2_, ⋯, *t*_*n*_ by *s*1, *s*2, ⋯, *sq*; and the matrix that shows the relationship between them is called the incidence matrix, which is denoted by *N*. *N* is an *n*∗*q* matrix whose elements are *N*_*i*_, if *t*_*i*_ = *s*_*j*_, and *N*_*ij*_ = 1; otherwise, *N*_*ij*_ = 0. If *t*_*i*_ is not identical, then *q* ≥ 2. Make *a*_*j*_ = *g*(*s*_*j*_), *j* = 1, 2, ⋯, *q*. Then the vector *g* to be estimated is (*a*_1_, *a*_2_, ⋯,*a*_*q*_。)′. Similarly, if *s*_1_ < *s*_2_ < ⋯<*s*_*q*_, and *a*_*j*_ = g(*s*_*j*_), then two matrices *Q* and *R* can be defined, except that *t*_l_, *t*_2_, ⋯, *t*_*n*_ should be replaced by *s*_1_, *s*_2_, ⋯, *s*_*q*_ and *K* = OR^−1^Q′, and then ∫*g*^′′(*s*)^2^^*ds* = *g*′*Kg*.

Use matrix notation to represent *S*_w_(*β*, *g*), then:

(3) $$\begin{array}{c} S_{w}\left(\beta ,g\right)={\left(Y-X\beta -Ng\right)}^{\prime }W\left(Y-X\beta -Ng\right)+\alpha {\text{g}}^{\prime }\text{Kg}. \end{array}$$

When *β* and *g* are solutions to the following partitioned matrix equation, the above formula takes a minimum.

(4) $$\begin{array}{c} \left[\begin{array}{cc} X^{\prime }WX & X^{\prime }WN\\ N^{\prime }WX & N^{\prime }WX+\alpha K \end{array}\right]\left(\begin{array}{c} \beta \\ g \end{array}\right)=\left[\begin{array}{c} X^{\prime }\\ N^{\prime } \end{array}\right]WY. \end{array}$$

### 3.2. Cross-Validation

Cross-validation is a method in which each observed value participates in both model establishment and model evaluation, in order to obtain the sum of squares of residuals (Prediction Residual Error Sum of Squares, PRESS), which reflects the disturbance error caused by the change of observation points. Finally, the total sum of squares of all residuals is obtained as the total sum of squares of residuals [17, 18]. The cross-validation method can be divided into

1. leave-one-out (LOO)
2. two batch cross-validation method
3. split-sample cross-validation method
4. random sample cross-validation method. For example, the batch cross-validation method, that is, *q* consecutive observations are detained as test data set each time, and the remaining observations are used to establish the model. When *Q* = 1, it is the truncated cross-validation method [19]. The larger the PRESS value is, the more unstable the model is. Finally, the number of extracted components is determined according to the principle of minimizing the sum of squares of predicted residuals

### 3.3. Experience Method

It is determined according to the cumulative contribution rate of components. Generally, extracted components explain most of the variation information of independent variables and dependent variables, such as 65%, 75%, and 80%. This method is similar to the determination of the number of principal components in principal component analysis. This method is simple and convenient but not accurate, and the accuracy of regression equation is not high [20].

### 3.4. Determination Method of Multiple Regression Equation

#### 3.4.1. Forward Selection Method

The forward selection method is to investigate the relationship between variables outside the equation and dependent variables and introduce the variables with the closest relationship into the equation one by one until there are no variables with significant relationship outside the equation to be introduced [21].

#### 3.4.2. Backward Elimination

That is, each variable is first included in the equation, and then the significance of the linear relationship between *X*′ and *Y* is judged, and the independent variables with no significant significance are removed from the equation one by one until all the independent variables contained in the formula have significant significance for *Y*.

#### 3.4.3. Stepwise Regression

This is a more reasonable and convenient method established on the basis of the previous two methods; that is, from the selected *m* independent variables, according to the size of the corresponding variable contribution of each variable, two-way cross is introduced and removed one by one for screening. Before and after an independent variable is selected or removed, a hypothesis test is performed to ensure that each time a new variable is introduced, only the independent variable that has a significant effect on *Y* is included in the equation. This is repeated until no independent variable with no significant effect can be removed from the equation, and no independent variable with significant effect can be selected outside the equation to achieve the optimal standard.

#### 3.4.4. Optimal Subset Regression Method

That is, from the subset regression equation of all possible combinations of all independent variables, the best one is selected according to some index (such as *R*^2^, modified *R*^2^, and *C*_*p*_). This method is foolproof, but when there are many independent variables, the calculation amount is very large (for example, there can be 2^m^-1 subset equation with m independent variables).

## 4. Outcome Analysis

### 4.1. Simulated Example Calculation

#### 4.1.1. The Research Group

All study samples were divided into age groups according to the age staging standard of pediatrics of the third edition of the eight-year program published by People's Medical Publishing House. It is divided into early childhood: 1- <3 years old; preschool age: 3- <6 years old; school-age: 6- <10 years old; and adolescence: 10 to 20 years old; there are four groups.

Forty pathological specimens of children with chronic tonsillitis were assigned to the tonsil group, and 50 pathological specimens were selected from 191 children with adenoid hypertrophy to the adenoid group by simple random sampling method. Ninety tonsil and adenoid specimens were divided into male group (*n* = 49) and female group (*n* = 41) according to sex. According to age grouping criteria, 90 cases of tonsil and adenoid pathological specimens were divided into infant group (*n* = 14), preschool age group (*n* = 20), school-age group (*n* = 25), and adolescence (*n* = 31). Ninety tissue specimens were divided into 1, 2, 3,… 90. After numbering, immunohistochemistry and in situ hybridization were performed [22].

#### 4.1.2. Simulation Example Calculation

A simulation example is given to illustrate the fitting effect of semiparametric model. In this example, *P* = 2, *n* = 60, *t* changes from 1 to 60, *x*1 ~ *n* (12.66, 2.57^2^), *x*2 ~ *N* (6.7, 1.87^2^), error terms *ε* are independent and distributed *N* (0, 5^2^), and *y* = 3.4*x*_1_ + 5.2*x*_2_ + 0.1(*t* − 30)^2^ + 30.2 + *ε*. A sample simulation data can be generated by SAS program, as shown in Tables 1 and 2.

Assuming that *y* is linearly dependent on *x*1 and *x*2, if the data is artificially fitted with a parametric linear model, the regression equation can be obtained: $\tilde{y}=49.0545+0.1282t+4.4925x_{1}-6.0078x_{2}$. Although the regression equation is meaningful (*P* ≈ 0.0005), the fitting effect is poor, SSE = 45494.6025, *R*^2^ = 0.2692, and the mean square error is 812.4037. It can be seen from Figure 2 that there is a conic trend between residual and *T*; that is, residual still contains useful regression information. If the semiparametric regression model is used for fitting, the calculated *α* value is 148.75, and the regression coefficients of *x*_1_ and *x*_2_ are 3.7976 and -5.2356, respectively. The test results were significant (*P* < 0.01), SSE = 980.6252, MSE = 19.2357, and *R*^2^ = 0.9842. The residual error of model fitting is shown in Figure 3. As can be seen from the above calculation results and Figure 3, the fitting effect of the semiparametric model has been greatly improved, and the relationship between *Y* and *T* has been correctly reflected [23, 24].

### 4.2. Comparison of EBER-Positive Rate in Different Tissues, Sex, and Age Groups

#### 4.2.1. Comparison of EBERs-Positive Expression Rate between Different Genders

In this study, paraffin-embedded tissue sections of 90 patients with chronic tonsillitis and adenoid hypertrophy were collected. EBERs were positive in 26 of the 49 male children, accounting for 53.06 of male children (26/49 cases); among 41 female children, 28 were EBERs positive, accounting for 68.29 of the female children (28/41cases). Set *χ*^2^ test, *χ*^2^ = 2.16, and *P* = 0.14 > 0.05 (see Table 3).

#### 4.2.2. Comparison of EBERs-Positive Rate in Different Age Groups

In 90 cases of chronic tonsillitis and adenoid hypertrophy of tonsils, there were 14 cases in the infant group, 20 cases in the preschool age group, 25 cases in the school-age group, and 31 cases in the adolescent group. The positive rate of EBERs was 42.86% (6/14 cases) in early childhood and 55.00 in preschool age (11/20 cases). The EBERs-positive rate was 60.00% in school-age group (15/20 cases) and 70.97 in adolescent group (22/31 cases). Set *χ*^2^ test, *χ*^2^ = 3.48, and *P* = 0.32 > 0.05 (see Table 4).

### 4.3. Analysis of T Lymphocyte Subsets in Children with Chronic Tonsillitis

The CD3 + T lymphocytes of 19 children with chronic tonsillitis in Epstein-Barr virus-positive group were 68.83 ± 3.941, CD4 + T cell were 31.23 ± 4.79, CD8 + T cell were 30.54 ± 5.54, and the ratio of CD4+/CD8+ was 1.02 ± 0.25. There was no statistical significance between these cells and the lymphoid subsets of children with chronic tonsillitis in the Epstein-Barr virus-negative group [25]. See Table 5 for details.

## 5. Conclusion

In this study, 40 cases of chronic tonsillitis in children and 50 cases of adenoid hypertrophy in children were examined for LMP1 and EBER. Based on regression equation, this paper focuses on semiparametric regression model method, cross validation method, empirical method, and multiple regression equation analysis of atypical data and gives the general method of analyzing this kind of data. The parameter estimation and hypothesis testing of the model were systematically studied. The T lymphocyte subsets in peripheral blood of 40 children with chronic tonsillitis were detected by flow cytometry, and the following conclusions were drawn:

The latent infection rate of adenoid hypertrophy EBV in children was higher than that of chronic tonsillitis in children.

The latent infection rate of adenoid hypertrophy EBV in children with chronic tonsillitis showed no significant difference between genders.

This study involves a relatively new field of statistics, many analytical methods are not perfect, and there is a lack of ready-made statistical software. In order to be convenient and practical, the obtained analysis methods need to be programmed in the future and then analyzed by examples to obtain satisfactory results through the program and verify their practicability.

## Figures and Tables

**Figure 1:** Regression equation flow.

**Figure 2:** Residuals of linear model fitting.

**Figure 3:** Residuals of semiparametric model fitting.

**Table 1:** Data list 1.

*t*	*x*_1_	*x*_2_	*ε*	*y*	$\hat{y}$
1	13.7573	9.0395	3.75143	117.821	113.7
2	15.052	7.3279	1.14067	122.813	122.411
3	8.6033	7.3862	0.23542	94.179	92.477
4	8. 6597	8.5354	-7.34831	75.51	81.595
5	15.260 7	4.0964	3.86252	127.148	124.918
6	12.7431	7.4814	-3.4369	88.786	92.752
7	16.268	6.4557	9.27355	114.115	106.738
8	10.168	5.2876	-3.75255	81.923	85.032
9	13. 2466	5.3008	0.40266	92.177	92.14
10	11.5926	5.5634	1.03347	81.719	80.133
11	6.7552	12.4906	-0.30367	24.013	21.325
12	12.956	8.818	-3.99901	56.798	60.147
13	11.1053	3.6854	-6.52679	71.167	76.288
14	7.7996	6.2757	-1.49224	48.193	46.746
15	16. 1694	6.3666	0.46688	75.036	74.903
16	12.5233	4.4313	1.40592	70.742	68.307
17	16.213	9.0616	-7.86257	47.241	55.469
18	12.7037	6.6083	4.72638	58.156	52.658
19	11.1916	6.9559	-0.50045	43.68	43.025
20	9.0719	10.1228	-2.09744	16.307	16.571
21	13.2374	8.2352	-2.20841	38.275	40.706
22	14.1714	6.0503	1.91203	55.233	54.373
23	12.148	5.0736	-5.52984	44.491	50.723
24	11.029	10.0753	3.65699	22.564	19.43
25	10.8887	8.3597	3.08169	29.333	27.203
26	15.014	5.5422	3.69035	57.719	57.095
27	14.0647	6.6078	2.63609	47.195	47.519
28	10.9326	6.8775	0.81989	32.828	33.939
29	12.3795	6.8564	3.39402	40.131	39.377
30	15.2033	11.4076	9.15392	31.726	26.192
31	12.7406	4.4082	3.07456	53.77	53.48
32	14.3541	4.9055	-2.34343	51.552	57.089
33	7.2211	7.3388	4.36714	21.857	17.452
34	12.2964	7.379	-0.13148	35.106	36.812
35	7.5594	5.2159	6.15973	37.439	30.556
36	13.783	6.797	0.10761	45.426	46.447
37	11.7396	6.5214	2.97025	44.074	40.832
38	9.2977	5.9949	-4.85962	32.179	35.232
39	8.6071	6.3306	-5.48525	29.16	32.042
40	11.2352	9.6646	-4.16542	23.979	26.075
41	13.8607	7.6723	-4.27133	45.259	48.329
42	13.6616	8.4751	-0.61364	46.365	45.577
43	14.8575	10.0036	-0.35908	45.238	44.672
44	11.3236	5.1932	-4.19473	57.101	59.337

**Table 2:** Data list 2.

*t*	*x*_1_	*x*_2_	*ε*	*y*	$\hat{y}$
45	13.0163	4.9998	-9.97231	60.984	70.019
46	11.2934	3.7157	0.90965	75.786	73.759
47	12.3691	4.0188	5.37863	85.636	80.071
48	13.1409	8.0467	9.53689	74.973	65.923
49	11.8286	7.1126	-8.29482	61.239	70.013
50	12.0206	5.9175	6.27481	86.574	81.372
51	9.9082	7.023	-3.72382	67.744	72.118
52	11.4828	8.8829	1.1973	72.648	73.099
53	7.1578	5.1667	-3.58128	76.989	81.040
54	16.1750	4.2811	6.46804	127.001	124.974
55	8.0296	3.9454	8.23395	107.718	100.957
56	12.2365	7.2613	-1.83271	99.812	104.805
57	14.5338	9.3725	2.89922	106.677	107.781
58	12.2149	8.6182	2.84722	108.163	108.284
59	14.1007	4.9623	8.82781	145.267	139.972
60	13.6661	48874	2.12864	143.379	144.101

**Table 3:** Expression rates of EBERs in children of different genders.

Sex	Cases	EBERs expression rates	
		Positive	Negative
Male	49	26 (53.06%)	23 (46.94%)
Female	41	28 (6829%)	13 (31.71%)

(note:*χ*^2^ = 2.16; *P* > 0.05).

**Table 4:** EBERs expression in different age groups.

Group	Cases	EBERs expression	
		Negative	Positive
Children's group	14	6 (42.86%)	8 (57.14%)
Preschool age group	20	11 (55.00%)	9 (45.00%)
School-age	25	15 (60.00%)	10 (40%)
Adolescence group	31	22 (70.97%)	9 (29.03%)

(Note:*χ*^2^ = 3.48; *P* > 0.05).

**Table 5:** Analysis of T lymphocyte subsets in children with EB-positive and negative Epstein-Barr virus chronic tonsillitis.

	CD3 + T(%)	CD4 + T(%)	CD8 + T(%)	CD4+/CD8+
EB virus positive	68.83 ± 394	31.23 ± 479	3054 ± 5.54	102 ± 0.25
EB virus negative	68.62 ± 390	32.82 ± 6.29	2993 ± 6.28	1 09 ± 0.27
*P* value	>0.05	>0.05	>0.05	>0.05

## Data Availability

The data used to support the findings of this study are available from the corresponding author upon request.
